The article "Tetramethylpyrazine and Paeoniflorin Synergistically Attenuate Cholesterol Efflux in Macrophage Cells via Enhancing ABCA1 and ABCG1 Expression" was published in 2022. Journal: Evid Based Complement Alternat Med.

# Tetramethylpyrazine and Paeoniflorin Synergistically Attenuate Cholesterol Efflux in Macrophage Cells via Enhancing ABCA1 and ABCG1 Expression

**DOI:** 10.1155/2022/4304790

**Published:** 2022-11-05

**Authors:** Jun Mei, Fengqin Xu, Qingbing Zhou, Ying Zhang, Jie Ji, Meng Li

**Affiliations:** ^1^Graduate School,, Beijing University of Chinese Medicine, Beijing, China; ^2^Institute of Geriatrics, Xiyuan Hospital, China Academy of Chinese Medical Sciences, Beijing, China

## Abstract

The formation of foam cells is a characteristic of the occurrence and development of atherosclerosis. ATP-binding cassette subfamily A1 and G1 (ABCA1 and ABCG1) and scavenger receptor B1 (SR-B1) play critical roles in promoting intracellular cholesterol efflux to high-density lipoprotein (HDL) or apolipoprotein A1 (apoA1). We attempted to test the effect of the tetramethylpyrazine-paeoniflorin pair (TP) on cholesterol outflow in foam cells derived from macrophages. In this study, RAW264.7 macrophages were treated with 80 mg/L oxidized low-density lipoprotein (ox-LDL) for 24 h to obtain foam cells. Then they were intervened with TP (tetramethylpyrazine 40 ug/ml plus paeoniflorin 80 ug/ml) for additional 24 h. The distribution of cholesterol in foam cells was evaluated by oil red O staining. The contents of total cholesterol (TC) and free cholesterol (FC) were assessed with commercial kits. Fluorescent imaging was observed with a fluorescent inverted microscope. The capacity of cholesterol efflux was measured with a fluorescent plate reader, and the transcript and protein levels of ABCA1, ABCG1, and SR-B1 were detected by Western blot and quantitative polymerase chain reactions (Q-PCRs). Cytokines in the medium were detected by ELISA and adjusted by total cellular proteins. The results showed that TP decreased ox-LDL-induced cholesterol deposition and foam cell formation by promoting cholesterol efflux to apoA1, which was related to the upregulation of ABCA1 and ABCG1. Moreover, TP decreased the secretion of ox-LDL-induced tumor necrosis factor alpha (TNF-*α*), interleukin 1 beta (IL-1*β*), and monocyte chemotactic protein-1 (MCP-1), an important profoam cell cytokine in atherosclerosis.

## 1. Introduction

Atherosclerosis is a pathological basis for ischemic cerebrovascular disease, coronary heart disease, and other cardiovascular diseases. Lipid accumulation in macrophage which is an early phase of atherosclerosis may result from uptake of excessive ox-LDL or impairment of cholesterol efflux capacity. Meanwhile, some inflammation reactions occur in the process with secretion of inflammatory factors [1].

In balanced lipid metabolism, HDL can transport cholesterol from foam cells and atherosclerotic plaques to the liver to synthesize bile, thereby reducing plaque size [2]. ABCA1 is a membrane protein that transports lipids across membranes to support HDL biosynthesis [3]. Likewise, ABCG1 has the ability to mediate cholesterol efflux to HDL or apoA1 and prevent intracellular lipid accumulation [4]. SR-B1 also facilitates the flow of cholesterol back to the liver from peripheral tissues, including macrophages [5].

The article "Tetramethylpyrazine and Paeoniflorin Synergistically Attenuate Cholesterol Efflux in Macrophage Cells via Enhancing ABCA1 and ABCG1 Expression" was published in 2022. Journal: Evid Based Complement Alternat Med.

It was reported that TNF-*α* and IL-*β* can augment inflammasome action to damage vessel endothelium, and increased atherosclerotic lesions in the arteries were related to concentration of these factors [6, 7]. MCP-1 (also referred to as chemokine C-C motif ligand 2, CCL2) is mainly expressed in inflammatory cells and endothelial cells. The expression levels of these cytokines are upregulated by ox-LDL-induced proinflammatory status and tissue injury [1].

Tetramethylpyrazine and paeoniflorin, two representative bioactive chemical compounds of Chuanxiong and Chishao, respectively, which are Chinese herbs, were reported that they had the abilities to attenuate atherosclerosis development [8, 9]. In the theory of traditional Chinese medicine, Chuanxiong and Chishao have synergistic effects in the treatment of thrombosis, atherosclerosis, inflammation, and other diseases [10]. Based on the above, it was hypothesized that tetramethylpyrazine and paeoniflorin have synergism to suppress lipid accumulation and inflammatory response.

In this study, we induced RAW264.7 macrophages to foam cells with ox-LDL and then assessed whether tetramethylpyrazine-paeoniflorin pair promotes the efflux of intracellular cholesterol via regulating ABCA1, ABCG1, or SR-B1 and decreasing the release of TNF-*α*, IL-*β,* and MCP-1.

## 2. Materials and Methods

### 2.1. Antibodies and Reagents

Tetramethylpyrazine and paeoniflorin were purchased from Kaimosi Biochemical Technology (Qingdao, China). Antiscavenger receptor class B type 1 antibody (SR-B1), anti-*β*-actin antibody, anti-ATP-binding cassette transporter A1 (ABCA1), and G1 (ABCG1) antibodies were purchased from Abcam (Cambridge, MA, USA). Goat antimouse IgG and HRP were purchased from Santa Cruz Biotechnology (Santa Cruz, CA, USA). Oil red O powder (ORO), apolipoprotein A1 (apoA1), and bovine serum albumin (BSA) were purchased from Sigma-Aldrich (St. Louis, MO, USA). High glucose Dulbecco's Modified Eagle's Medium (DMEM) was purchased from HyClone (Thermo Fisher Scientific, Waltham, MA, USA). High glucose DMEM Phenol Red (DMEMWPR) and fetal bovine serum (FBS) were purchased from Gibco (Thermo Fisher Scientific, Waltham, MA, USA). Oxidized low-density lipoprotein (ox-LDL) was purchased from Yiyuan Biotech (Guangzhou, China). NBD-cholesterol and penicillin-streptomycin-neomycin (PSN) antibiotic mixture was purchased from Thermo Fisher Scientific (Waltham, MA USA).

The article "Tetramethylpyrazine and Paeoniflorin Synergistically Attenuate Cholesterol Efflux in Macrophage Cells via Enhancing ABCA1 and ABCG1 Expression" was published in 2022. Journal: Evid Based Complement Alternat Med.

### 2.2. Cell Culture

Raw264.7 cell line was obtained from the Cell Bank of the Chinese Academy of Sciences (Beijing, China). Cells were maintained in DMEM (4 mM L-glutamine, 4.5 g/L glucose) containing 10% FBS (50 U/ml-50 ug/ml-100 ug/ml), PSN at 37°C under 5% CO2, and passaged every 2-3 d. They were treated with 80 mg/L ox-LDL for 24 h to induce differentiation into foam cells after inoculating 2 ml RAW264.7 cell suspension (about 100 thousand cells) into 6-well plates. The treatment concentrations are derived from the cell experiment data of our research group [11].

### 2.3. Oil Red O Staining

The distribution of cellular lipid accumulation was evaluated by ORO staining in RAW264.7 cells. RAW264.7 cells were cultured in 96-well plates, and 80 mg/mL ox-LDL was added for 24 h and then tetramethylpyrazine or paeoniflorin or tetramethylpyrazine-paeoniflorin pair was added and incubated for another 24 h. Finally, cells were fixed and stained with ORO and observed on an inverted microscope (Leica, Wetzlar, Germany).

### 2.4. Cellular Cholesterol Assay

Intracellular total cholesterol (TC) and free cholesterol (FC) levels were detected by using cholesterol assay kits, an enzymatic assay technique, (Applygen Technologies, Beijing, China) according to the manufacturer's protocol.

### 2.5. Fluorescent Imaging

The RAW264.7 cells were seeded in 12-well plates (Costar, Corning, NY, USA) for 24 h. Then, they were loaded with 50 ug/ml ox-LDL and 5 ug/ml NBD-cholesterol in serum-free medium containing 0.2% (w/v) BSA for another 24 h to be transformed into foam cells with fluorescent. Then, the cells were washed twice with DMEMWPR, and cholesterol efflux proceeded for 24 h at 37°C in 0.5 ml DMEMWPR containing nothing, 40 ug/ml tetramethylpyrazine, 80 ug/ml paeoniflorin, 40 ug/ml tetramethylpyrazine plus 80 ug/ml paeoniflorin, and 15 ug/ml lipid-free human apoA1, respectively. At the end of this treatment, the medium was collected and the cells were washed twice with DMEMWPR again. Subsequently, the fluorescent imaging of cells in DMEMWPR was observed on a fluorescence inverted microscope (Axio Observer 3, ZEISS, Germany). After observation, the fluorescence intensity of cell lysate was measured.

### 2.6. Cholesterol Efflux

The capacity of cholesterol efflux was tested with NBD-cholesterol in RAW264.7 macrophages. The cells were handled as above. At the end of this incubation, the medium was collected and centrifuged at 13,000 rpm for 10 min to remove sediment. Cells were lysed with 0.5 ml of 0.1% Triton X-100 for 30 min, and the supernatant was collected and centrifuged at 13,000 rpm for 10 min [12]. The medium and cell lysate were detected for fluorescence intensity in 96-wellclear-bottom black plates (Costar, Corning, NY, USA) by fluorometry (Tecan Spark 10M; excitation 469 nm, emission 537 nm). The rate of cholesterol efflux was analyzed as follows: fluorescence intensity in the medium/(fluorescence intensity in the medium + fluorescence intensity in the cell lysate).

The article "Tetramethylpyrazine and Paeoniflorin Synergistically Attenuate Cholesterol Efflux in Macrophage Cells via Enhancing ABCA1 and ABCG1 Expression" was published in 2022. Journal: Evid Based Complement Alternat Med.

### 2.7. Western Blot Analysis

After cells were lysed with 0.1% Triton X-100, the concentrations of total protein were examined with BCA Protein Assay Kits (Beyotime Biotechnology, Shanghai, China). After normalization, equal total proteins were applied to 8% (ABCA1), 10% (ABCG1), and 12% (SR-B1) SDS-PAGE gels. Separated proteins by separating the gel were transferred onto PVDF membranes (Millipore, MA, USA). Then, the membranes were blocked with free-fat milk in TBS at 4°C for 1.5 h and incubated with primary antibodies for ABCA1 (1 : 300 dilution), ABCG1 (1 : 500 dilution), SR-B1 (1 : 500 dilution), and *β*-actin (1 : 3000 dilution), subsequently. At last, the membranes were incubated with HRP-conjugated antibodies for 2 h at room temperature.

### 2.8. Q-PCR

Total RNA was extracted from macrophages with an RNeasy kit (Tiangen Biochemical technology), and cDNA was prepared with a cDNA reverse transcription kit (Takara). mRNA expression was measured using the Q-PCR system (Applied Biosystems) with TaqMan primers for mouse ABCA1, ABCG1, and SR-B1. RT-qPCR was conducted in a 20 *μ*l mixture, including 2 *μ*l of the cDNA templates, 10 *μ*l × UltraSYBR Mixture (CoWin), 0.8 *μ*l of the 10 *μ*M sense and antisense primers, and 6.4 *μ*l ddH2O, using Line Gene 9600 Plus (Bioer Technology, Hangzhou, China). The RT-qPCR conditions were as follows: 10 min at 95°C, followed by 45 cycles between 95°C for 15 s and 60°C for 60 s. Fold changes of mRNA expression were calculated by the 2^−ΔΔCT^ method using mouse *β*-actin as an internal control for mRNA expression. All fold changes are compared to the control cells. The sequences of the primers were as follows in Table 1.

### 2.9. Statistical Analysis

All data are presented as means ± SD. Results were analyzed by Student's *t*-test and one-way ANOVA analysis by using GraphPad Prism 6.01 software. A *P*-value less than 0.05 was considered significant.

## 3. Result

### 3.1. Tetramethylpyrazine-Paeoniflorin Pair Attenuates RAW264.7 Macrophage Foam Cell Formation

Tetramethylpyrazine and paeoniflorin were found with good cholesterol reverse transport activity [9, 10]. The respective structure of tetramethylpyrazine and paeoniflorin is shown in Figures 1(a) and 1(b). At first, the proliferation activity of foam cells derived from RAW264.7 cell was measured by CCK-8 after treating 24 h with different concentrations of tetramethylpyrazine or paeoniflorin. The results showed that the two drugs below 80 ug/ml concentrations had no significant effect on the proliferation activity of foam cells (Figure 1(c)). To detect the synergetic effect of TP on foam cell formation, Raw264.7 cells were treated with 80 ug/ml ox-LDL for 24 h and then treated in the presence of tetramethylpyrazine and/or paeoniflorin for additional 24 h. ORO staining showed that the Raw264.7 cells induced by ox-LDL presented a foam cell model characterized by lots of lipid droplets and foamy morphologic (Figure 1(f)). Compared with foam cells in the model group, ORO staining showed that the lipid accumulation was decreased after 24 h treatment with TP (Figure 1(f)). Based on the references, we know that the biological effect of tetramethylpyrazine is only positively correlated with the concentration within a certain range, which is why T80 has a weaker effect than T40, although both T40 and T80 reduce total cholesterol. Because of the shooting conditions, the background of the oil red stained picture is variegated. If insisting on quantitative analysis, it is very likely to cause data error. Moreover, the intracellular cholesterol outflow is the main therapeutic effect index. Therefore, quantitative analysis is not conducted in this paper.

The article "Tetramethylpyrazine and Paeoniflorin Synergistically Attenuate Cholesterol Efflux in Macrophage Cells via Enhancing ABCA1 and ABCG1 Expression" was published in 2022. Journal: Evid Based Complement Alternat Med.

The TC and FC in foam cells treated by them were also determined. Tetramethylpyrazine itself had an ability, which was the highest at 40 ug/ml, to promote cholesterol outflow from foam cells, and TP, which is tetramethylpyrazine of 40 ug/ml plus paeoniflorin of 80 ug/ml, significantly facilitated more cholesterol outflow. Compared with the control group, TP clearly reduced the levels of intracellular total cholesterol (Figures 1(d) and 1(e)). The quantitative analysis further found that 24 h TP-treated foam cells decreased almost 40% of total cholesterol content and 50% of free cholesterol levels than the foam cells cultured in free media (Figures 1(d) and 1(e)). Based on these data, it was suggested that TP can reduce intracellular lipid accumulation in foam cells derived from RAW264.7 macrophages.

### 3.2. Tetramethylpyrazine-Paeoniflorin Pair Improved NBD-Cholesterol Efflux from Foam Cells

To investigate whether TP promotes cholesterol efflux from foam cells, the NBD-cholesterol as a marker was observed to cholesterol outflow in foam cells, and 15 ug/ml apoA1 was added as the acceptor in DMEMWPR.  Figure 2(a) shows that TP significantly increased cholesterol efflux from foam cells. Fluorescent imaging has shown that 24 h-TP treatment decreased lipid deposition compared to ox-LDL group; however, the intracellular fluorescence intensity looks even lower in the “ox-LDL + apoAI” group than that in the “ox-LDL + *T* + apoAI” group or the “ox-LDL + *P* + apoAI” group because of the smaller cell density (Figure 2(b)). These data showed that lipid accumulation was effectively inhibited by TP in RAW264.7 cells.

The article "Tetramethylpyrazine and Paeoniflorin Synergistically Attenuate Cholesterol Efflux in Macrophage Cells via Enhancing ABCA1 and ABCG1 Expression" was published in 2022. Journal: Evid Based Complement Alternat Med.

### 3.3. Tetramethylpyrazine-Paeoniflorin Pair Weakens Ox-LDL Induced Proinflammation Status of Raw 264.7 Cells

Cytokines can be detected in all phages of the atherosclerosis process and significantly affect the occurrence and development of atherosclerosis. Many cytokines including TNF-*α*, IL-1*β,* and MCP-1 are expressed in atherosclerotic plaques, which impact foam cell formation and the progression of atherosclerosis [13, 14]. To examine whether TP affected the secretion of cytokines in ox-LDL-induced foam cells, the medium was collected for detection. The analysis results showed that TNF-*α*, IL-1*β,* and MCP-1 were significantly increased in macrophage foam cells which may promote foam cell formation [15–17], but they were obviously decreased after 24 h-TP treatment (Figures 2(c)–2(e)).

### 3.4. Tetramethylpyrazine-Paeoniflorin Pair Improved the Expression of ABCA1 and ABCG1

We tested whether TP improved cholesterol efflux to lipid-poor apoA1, a lipid transport mediated by ABCG1, SR-B1, or ABCA1, respectively. Intracellular cholesterol analysis and fluorescent imaging showed that TP treatment indeed promoted cholesterol efflux from foam cells to apoA1 in DMEMWPR (Figures 2(a) and 2(b)). In consistent with this observation, we found TP facilitated ABCG1 and ABCA1 expression at transcript as well as protein levels, and only SR-B1 expression at transcripts, but the levels of SR-B1 proteins were not obviously increased (Figures 3(a)-3(g)), which was reported to facilitate the cholesterol outflow from macrophages [5]. These data suggested that TP may specifically improve ABCA1- and ABCG1-mediated cholesterol efflux, not SR-B1 pathway.

## 4. Discussion

The cholesterol efflux ability of macrophages is strongly negatively correlated with carotid intima media thickness and the possibility of coronary heart disease [18]. Cholesterol depletion due to the uptake of oxidized lipids leads to cholesterol accumulation and foam cell formation, while foam cells form fatty streaks and plaques in the late stage of atherosclerosis [19]. In addition, there are many cytokines which are secreted in the process of foam cell formation, so atherosclerosis is also seen as a chronic inflammatory process [14].

The first step of RCT is the outflow of cholesterol from foam cells to apoA1 for HDL formation, which is mainly mediated by ABCA1, ABCG1, or SR-B1, especially ABCA1 accounting for the majority of the total in cholesterol efflux [20–22]. Both ABCA1 and ABCG1 are members of the ATP-binding cassette (ABC) transporter superfamily which transport intracellular cholesterol across membrane to extracellular [4, 23]. The absence of ABCA1 gene will result in Tangier disease characterized with lipid metabolism disorder and absent HDL levels in human [24]. ABCG1 can also promote intracellular cholesterol efflux to HDL. When ABCG1 gene was silenced, large amounts of lipid were deposited in the tissues of the liver and macrophages of mice fed with a high-fat diet. In contrast, overexpression of ABCG1 can protect macrophages and tissues from dietary fat induced lipid accumulation [4]. SR-B1 is a glycoprotein widely expressed in multiple tissues, such as the liver, macrophages, adipocytes, and other cellular tissues [22]. SR-B1 regulates intracellular FC transport by selective uptake of cholesterol esters from HDL-C and mediating cholesterol outflow from macrophages to mature HDL particles [25].

The article "Tetramethylpyrazine and Paeoniflorin Synergistically Attenuate Cholesterol Efflux in Macrophage Cells via Enhancing ABCA1 and ABCG1 Expression" was published in 2022. Journal: Evid Based Complement Alternat Med.

Our previous studies indicated that Xiongshao capsule containing tetramethylpyrazine and paeoniflorin, which could reduce the serum TC, FC, and myeloperoxidase (MPO) levels in aorta cells of AS rabbits, prevented atherosclerosis [26, 27]. However, the underlying molecular and biological mechanisms remain unclear. In this study, we treated foam cells with tetramethylpyrazine and/or paeoniflorin, two typical bioactive chemical compounds of Xiongshao capsule, and our results showed that TP could promote cholesterol efflux from foam cells and reduce the intracellular lipid deposition in macrophages. In addition, TP facilitated the expression of ABCG1 and ABCA1 both at relative mRNA and protein intensity, only SR-B1 at transcript levels. Furthermore, we thought that TP increased cholesterol efflux to apoA1 and reduced lipid accumulation in macrophages based on the upregulation of ABCA1 and ABCG1, displaying a protective effect of TP on preventing macrophages from turning into foam cells. Previous studies have shown that ligustrazine can upregulate the expression of ABCA1 and ABCG1 and promote the cholesterol efflux of foam cells. However, in this study, we also found that ligustrazine can promote the cholesterol efflux of foam cells, but it failed to significantly upregulate ABCA1 and ABCG1, which is not completely consistent with the previous research results. It is considered that it is related to the difference in experimental conditions, including the difference in drug source and intervention concentration [28–30].

The article "Tetramethylpyrazine and Paeoniflorin Synergistically Attenuate Cholesterol Efflux in Macrophage Cells via Enhancing ABCA1 and ABCG1 Expression" was published in 2022. Journal: Evid Based Complement Alternat Med.

Atherosclerosis is considered a chronic inflammatory process of the arteries which is influenced by a variety of cytokines produced by atherosclerotic plaques and foam cells. Intracellular lipid metabolism can be affected with some inflammatory cytokines including TNF-*α*, IL-1*β,* and MCP-1. The levels of IL-1*β* and TNF-*α* were upregulated at the site of atherosclerotic plaque [17]. IL-1*β* induces own expression and activation of some proinflammatory cytokines like MCP-1 [6, 31]. TNF-*α* can increase the intake of oxidized LDL, induce macrophages to transform into foam cells, accelerate the apoptosis of foam cells, and promote the formation of atherosclerotic plaques [14, 32]. In addition, TNF-*α* can upregulate the expression of MCP-1 and inhibit the expression of scavenger receptor A [33]. Atherosclerotic plaques are smaller mouse models lacking MCP-1 or its receptor [15, 34]. Moreover, some cytokines have been reported to directly affect the level of ABC transporters. Studies have shown that TNF-*α* and IL-1*β* can reduce the transcriptional levels of ABCA1 and ABCG1 [35]. In our experiments, TP inhibited TNF-*α*, IL-1*β,* and MCP-1 levels, suggesting that the antiatherosclerosis ability of TP may be related not only to reverse cholesterol transport but also to its anti-inflammatory potential.

It was reported that increased expression of liver *X* receptor alpha (LXR*α*) through peroxisome proliferator-activated receptor gamma (PPAR*γ*) can inhibit the secretion of IL-1*β* and TNF-*α*, but inhibition of LXR*α* expression canceled the inhibitory function [36]. Likewise, IL-1*β* and TNF-*α* can decrease the activation of PPAR*γ* and LXR*α* [37]. A study provided evidence that activation of PPAR*γ* can lead to a complete inhibition of MCP-1 at the gene and protein levels [38]. PPAR*γ* promotes the expression of ABCA1 and ABCG1 and cholesterol removal from foam cells mediated by LXR*α*, and PPAR*γ*-LXR*α*-ABCA1/ABCG1 is a pathway which regulates the transmembrane transport of intracellular lipids [39, 40]. Our data found that TP can upregulate the expression of ABCA1 and ABCG1 and inhibit the generation of TNF-*α*, IL-1*β,* and MCP-1. It was speculated that the abovementioned results were carried out by TP through activating PPAR*γ*/LXR*α* pathway which we would explore in our future work.

## Figures and Tables

**Figure 1:** TP reducing intracellular lipid accumulation in foam cells derived from RAW264.7 macrophages. (a) The chemical structure of tetramethylpyrazine. (b) The chemical structure of paeoniflorin. (c) The proliferative activity of foam cells derived from RAW264.7 macrophages treated with tetramethylpyrazine (5, 10, 20, 40, and 80 ug/ml) or paeoniflorin (5, 10, 20, 40, and 80 ug/ml). (d) Levels of TC in RAW264.7 macrophages treated with control (high glucose DMEM with 10%FBS) or ox-LDL (80 ug/ml) or tetramethylpyrazine (5, 10, 20, 40, and 80 ug/ml) or tetramethylpyrazine-paeoniflorin pair (T40 plus P5, 10, 20, 40, and 80 ug/ml). (e) Levels of TC in RAW264.7 macrophages treated with above as (d). (f) ORO staining photographs of RAW264.7 cells induced by 24 h ox-LDL treated with tetramethylpyrazine and/or paeoniflorin for 24 h (200× magnification). Four independent experiments have shown similar results. Data were shown with MD ± SEM (*n* = 4, ^*∗*^*P* < 0.05 vs. control, ^*∗∗*^*P* < 0.01 vs. control; ^#^*P* < 0.05 vs. ox-LDL, ^##^*P* < 0.01 vs. ox-LDL).

The article "Tetramethylpyrazine and Paeoniflorin Synergistically Attenuate Cholesterol Efflux in Macrophage Cells via Enhancing ABCA1 and ABCG1 Expression" was published in 2022. Journal: Evid Based Complement Alternat Med.

**Figure 2:** Tetramethylpyrazine-paeoniflorin pair improved NBD-cholesterol outflow from foam cells and ox-LDL induced proinflammation status of Raw 264.7 cells. (a) and (b) RAW264.7 cells were treated with 50 ug/ml ox-LDL and 5 ug/ml NBD-cholesterol in serum-free medium containing 0.2% (w/v) BSA for 24 h and then treated with control (high glucose DMEM with 10%FBS) or ox-LDL (80 ug/ml) or tetramethylpyrazine-paeoniflorin pair (T40 plus P5, 10, 20, 40, and 80 ug/ml) for additional 24 h Then, the capacity of cholesterol efflux was analyzed by using a fluorescence microplate reader. The efflux rate is calculated with the formula: fluorescence intensity in the medium/(fluorescence intensity in medium + fluorescence intensity in the cell lysate). ((c)-(e)) The foam cells were treated with tetramethylpyrazine and/or paeoniflorin, and profoam cytokines were detected. All data were shown as MD ± SEM of four independent experiments. (*n* = 4, ^*∗*^*P* < 0.05 vs. control, ^*∗∗*^*P* < 0.01 vs. control; ^#^*P* < 0.05 vs. ox-LDL, ^##^*P* < 0.01 vs. ox-LDL;^Δ^*P* < 0.05 vs. apoA1, ^ΔΔ^*P* < 0.05 vs. apoA1).

**Figure 3:** Tetramethylpyrazine-paeoniflorin pair increased cholesterol efflux mediated by ABCA1 and ABCG1 in foam cells. ((a)-(d)) The impact of tetramethylpyrazine and/or paeoniflorin on the relative protein intensity of cholesterol transporters in foam cells. ((e)-(g)) The relative mRNA intensity of cholesterol transporters in foam cells treated with tetramethylpyrazine and/or paeoniflorin. All data were shown as MD ± SEM of three independent experiments. (*n* = 3, ^*∗*^*P* < 0.05 vs. control, ^*∗∗*^*P* < 0.01 vs. control; ^#^*P* < 0.05 vs. ox-LDL, ^##^*P* < 0.01 vs. ox-LDL).

**Table 1:** Primer sequences used in the study.

Name of the primer	Primer sequence (5' to 3')	Size (bp)
ABCA1 sense	GCTCTCAGGTGGGATGCAG	81
ABCA1 antisense	GGCTCGTCCAGAATGACAAC	
SR-BI sense	TTTGGAGTGGTAGTAAAAAGGGC	71
SR-BI antisense	TGACATCAGGGACTCAGAGTAG	
ABCG1 sense	CGAAGCCAAGAAGGTCCTGAG	283
ABCG1 antisense	CAGAGCAGCGAACAGCACAA	
*β*-actin sense	GCCTTCCTTCTTGGGTAT	97
*β*-actin antisense	GGCATAGAGGTCTTTACGG	

The article "Tetramethylpyrazine and Paeoniflorin Synergistically Attenuate Cholesterol Efflux in Macrophage Cells via Enhancing ABCA1 and ABCG1 Expression" was published in 2022. Journal: Evid Based Complement Alternat Med.

## Data Availability

Some or all data, models, or code generated or used during the study are available from the corresponding author by request.
